This article has been retracted.

# Inhibition of TLR4 Suppresses the Inflammatory Response in Inflammatory Bowel Disease (IBD) by Modulating the PDK1-Induced Metabolism Reprogramming via a m6A-Denpendent Manner

**DOI:** 10.1155/2022/1335562

**Published:** 2022-07-04

**Authors:** Jing Wang, Jing Huang, Liang Fang

**Affiliations:** Department of Digestive Medicine, Huanggang Central Hospital, Hubei Province Huanggang City 438000, China

## Abstract

**Objective:**

To investigate the role of TLR4 and PDK1 genes in IBD.

**Methods:**

The DSS mouse model was established by inducing BALB/C with 5% DSS solution. The behavior of DSS mice was detected, and the m6A modification was detected by m6A methylation chip. At the same time, the expressions of TLR and PDK1 were detected by fluorescence real-time quantitative PCR.

**Results:**

The results showed that the model of dextran sodium sulfate colitis in mice was successful, and the colon membrane of mice had obvious naked eye inflammation. Through comparison, it was found that there were differences in m6A modification between the blank group and the model group, and compared with the blank group, the expression of PKD1 in DSS group was significantly reduced and the expression of TLR4 was significantly increased.

**Conclusion:**

TLR4 inhibition inhibits the inflammatory response in inflammatory bowel disease (IBD) in a m6A-dependent manner by regulating PDK1-induced metabolic reprogramming.

## 1. Introduction

Inflammatory bowel disease (IBD) is a chronic nonspecific inflammatory disease of the intestine with unclear etiology, mainly including ulcerative colitis (UC) and Crohn's disease (CD). Many factors such as heredity, environment, infection, and immunity are involved in the pathogenesis, among which intestinal inflammation and immune dysfunction play an important role [1]. Genetic susceptibility can partly explain the differences in the pathogenesis of IBD. With the progress of molecular biology technology, epigenetics, as one of the ways to regulate gene expression, has been gradually explored and established in IBD, and its relationship with IBD is particularly close [2]. The mature research is DNA methylation. The changes of DNA methylation modification are suggested in the peripheral blood or colon tissue of IBD patients [3, 4]. RNA methylation is a newly discovered epigenetic modification of RNA in recent years, which can regulate the expression of messenger RNA (mRNA). The most common modification method is N6-methyladenine (m6A). There are more and more studies on RNA methylation and diseases, including tumors, nervous system diseases, obesity, and immune response, but the relationship with IBD is not clear.

M6A modification involves almost all aspects of RNA metabolism. It can affect the expression level of mRNA and protein by affecting mRNA precursor splicing, mRNA transport, and degradation and regulating mRNA translation, which is the basis for speculating that m6A is involved in IBD inflammation and immune regulation. Therefore, this study explored the relationship between PDK1-induced metabolic reprogramming and m6A.

Dendritic cells (DCS) are antigen-presenting cells that coordinate the body's protective immunity and immune tolerance. Their abnormal migration and activation exacerbate intestinal mucosal inflammation [5]. It was found that m6A methylation promoted the activation of DCS, the level of m6A modification increased during the maturation of DCS, and the transcription and translation of mRNA expressing CD40, CD80, and toll/IL-1 receptor adaptor protein increased after m6A modification, promoting toll-like receptor (TLR) 4/NF-1*κ*B pathway mediated inflammatory factor production and T cell activation [6]. At the same time, some studies have shown that there is a close relationship between PDK1 and TLR4. Therefore, this study studied the inhibition of TLR4 by regulating PDK1-induced metabolic reprogramming and inhibiting the inflammatory response in inflammatory bowel disease (IBD) in a m6A-dependent manner.

## 2. Methods

### 2.1. Establishment of DSS Rat Colitis Model

Dextran sodium sulfate (DSS) with a molecular weight of 5000 was dissolved in distilled water and prepared into a 5% DSS solution. BALB/c mice were allowed to drink freely for 7 days to establish a mouse model of acute colitis. From the date of modeling, the weight, activity, eating, stool characteristics, and stool blood of mice were observed every day (fecal occult blood was detected by benzidine method), and the disease activity index (DAI) of mice was scored [7].

### 2.2. Colon Score

After 7 days from the date of modeling, the mice were killed by neck breaking and dislocation method and laparotomy, the anus was taken to the colon of the first part of the ileus, and the colon was cut longitudinally along the edge of the mesentery. After washing with precooled normal saline, the general morphology of the intestine was observed under the anatomical microscope [8].

### 2.3. m6A-Modified Methylation Chip through Junction

Two groups of intestinal tissue samples were taken during enteroscopy biopsy, washed with 0.9% sodium chloride solution, put into the EP tube containing RNA preservation solution, cooled in liquid nitrogen, and stored in the refrigerator at -80°C. The changes of m6A modification were detected by m6A methylation chip [9].

### 2.4. RT-PCR Detection

After extracting total RNA from mouse colon tissue, measure the absorbance (*A*) values at 260 nm and 280 nm under the spectrophotometer, take RNA samples with a260/A280 of 1.8~2.0, and synthesize cDNA according to the instructions of cDNA first-strand synthesis kit. The real-time reverse transcription polymerase chain reaction was carried out by using the steps described in the instructions of the fluorescence quantitative detection kit, and the reaction was carried out by PCR instrument. Three multiple wells were made for the same gene real-time RT-PCR corresponding to each sample [10].

### 2.5. Statistical Analysis

All experimental data in this study are expressed as the mean ± standard deviation. Two groups of data were compared by an independent sample *t*-test, and multiple groups of data were compared by one-way ANOVA. All statistical analyses were completed by GraphPad prism 8 software. *P* < 0.05 was considered statistically significant.

## 3. Results

### 3.1. Observation on General State of Mice

On the first day after drinking DSS water, each mouse in the model group gained weight, drank more water, and ate more food. On the third day after drinking DSS, the weight of mice decreased, their hair was dull, their drinking and eating decreased significantly, their mucus was sparse, and some of them were positive for occult blood in stool, and the symptoms were gradually aggravated; On the 4TH-5TH day after drinking DSS water, some mice had more serious symptoms, such as bloody stool, obvious weight loss, loose hair, laziness, and mental depression. Mice died on the 6th day of modeling. By the end of the experiment, two mice in the model group died. During the experiment, the mice in the normal control group had normal stool, weight gain, shiny hair, diet, activity, and mental state and no death.

### 3.2. Change of Stool Characteristics

In the course of administration, about 2 mice in the model group had loose stool on the second day after administration, 4 mice had yellow green or light yellow loose stool or semi loose stool on the third day, of which 3 mice had positive occult blood in stool, 2 mice had bloody stool and blood in anus on the fourth day, and then, the symptoms gradually worsened. At least 3 mice had blood in anus during observation. Combined with various scores, it was proved that the modeling was successful.

### 3.3. Weight Change

As shown in Table 1, there was no significant difference in the weight of mice in each group before the experiment. After the experiment, the weight of mice in the model group drinking DSS decreased significantly, and the weight difference (the difference between after the experiment and before the experiment) was significantly different from that of mice in the normal control group.

### 3.4. The Expressions of m6A

Compared with the blank group, there were 11 m6A modifications with different m6A in the DSS group, including 7 modifications upregulated and 4 modifications downregulated.

### 3.5. The Expressions of PDK1 and TLR4 Were Detected by RT-PCR

Compared with the blank group, the expression of PDK1 was downregulated and the expression of TLR4 was significantly upregulated in Figures 1 and 2.

## 4. Discussion

Inflammatory bowel disease (IBD) is a kind of chronic recurrent nonspecific intestinal inflammatory lesions, including ulcerative colitis (UC), and Crohn's disease (CD). Its pathogenesis is not clear [11–14]. The application of animal model plays an important role in the in-depth study of its pathogenesis. Dextran sodium sulfate (DSS) induction is one of the most commonly used animal models of colitis. It can be seen from this experiment that BALB/c mice began to lose weight, have dull hair, significantly reduce drinking and eating, and have loose mucus, and some have positive fecal occult blood after 3 days of free drinking 5% dextran sodium sulfate (DSS). On the 4th day after drinking DSS, some mice had bloody stool, obvious weight loss, loose hair, lazy movement, and mental depression. Later, with the time of drinking 5% dextran sodium sulfate (DSS) gradually prolonged, the above manifestations gradually aggravated. The above results also prove that the colitis model of dextran sodium sulfate (DSS) in mice is successful, and it is verified again that BALB/c mice can drink 5% DSS freely, which is one of the better animal models to study IBD [15, 16].

Intestinal mucosal inflammation and abnormal immune system are the key mechanisms of IBD [17, 18]. Through RNA sequencing and function enrichment analysis, the differentially expressed genes after mettl3 knockout are closely related to the inflammatory response signal pathway [19, 20]. M6A can regulate the expression of key factors involved in the process of innate and adaptive immunity by regulating RNA splicing, stability, and other mechanisms, affect the function of immune cells, and cause abnormalities in the process of immune regulation. Innate immune response is the first defense line of intestinal mucosal immunity, including dendritic cells, macrophages and other immune cells, interleukin (IL), and tumor necrosis factor *α* (tumor necrosis factor-*α* (TNF*α*)), and other cytokines, involving nuclear factor-*κ*B (nuclear factor *κ*B (NF-*κ*B)). A series of signal transduction factors such as MAPK, jakin/kinase, and Jan signal kinase are activated. A variety of nonspecific inflammatory mediators and proinflammatory cytokines were significantly increased in the colon of IBD patients. Dendritic cells (DCS) are antigen-presenting cells that coordinate the body's protective immunity and immune tolerance. Their abnormal migration and activation exacerbate intestinal mucosal inflammation [21–27]. It was found that m6A methylation promoted the activation of DCS, the level of m6A modification increased during the maturation of DCS, and the transcription and translation of mRNA expressing CD40, CD80, and toll/IL-1 receptor adaptor protein increased after m6A modification, promoting toll like receptor (TLR) 4/NF-1*κ*B pathway mediated inflammatory factor production and T cell activation [28]. M6A can be involved in regulating the migration of DCs from the periphery to lymph nodes. Liu et al. [29] found that a noncoding RNA (LNC-DPF3) has m6A modification. After m6A demethylation, the expression of LNC-DPF3 increases, which inhibits DCS migration and inflammatory response by affecting the glycolysis pathway mediated by hypoxia inducible factor-1.

PIP3 produced by PI3K is considered to be the second messenger of insulin. PIP3 cannot directly activate Akt/PBK but can aggregate Akt/PBK to the cell membrane and change the results. PI3K and PDK1 form upstream and downstream pathways in cells [30, 31]. They are closely related as the key links of their respective metabolic regulation. PIP3 produced by PI3K can activate PDK1 and aggregate Akt protein on cell membrane. Under the action of PDK1, it phosphorylates serine phosphorylation site 437 (ser437) and threonine phosphorylation site 308 (thr308) on Akt protein and activates Akt signal pathway [32].

As an important pattern recognition receptor, TLRs can sense the existence of pathogenic microorganisms and produce immune inflammatory response in time by recognizing the corresponding pathogen related molecular patterns (PAMPs), and finally activate the acquired immune system [33]. The important role of TLRs in the body's immune response has been recognized by many scholars. Recently, it is also considered to be a kind of substance of intestinal immune response, which also plays an important role in maintaining intestinal membrane homeostasis. At present, some scholars believe that the environment (intestinal flora, intestinal mucosal barrier, food antigen, etc.), the body's immune response, and genetic susceptibility as a whole jointly affect the function of TLRs in intestinal membrane expansion. When the mutual regulation relationship between the three is unbalanced, it will lead to abnormal TLR signal transduction and eventually contribute to the occurrence and development of acute and chronic inflammation of colon in IBD [34]. Some scholars also believe that IBD is an imbalance of immune tolerance of intestinal immune system to normal intestinal flora caused by changes in environmental factors in susceptible individuals [33–35]. This experiment found that the expression of TLR4 was significantly increased in the colon of DSS mice.

## 5. Conclusion

The expression of TLR4 and PKD1 genes in the colonic membrane of DSS colitis mice is correlated and consistent, suggesting that they may play a synergistic role in the occurrence and development of DSS induced colitis in mice and jointly promote and aggravate the occurrence and persistence of inflammatory response. We speculate that the inflammatory response induced by TLR4 in IBD is inhibited by m6a.

## Figures and Tables

**Figure 1:** The expressions of PDK1 were detected by RT-PCR.

**Figure 2:** The expressions of TLR4 were detected by RT-PCR.

**Table 1:** Comparison with the difference of weight, length of colon, and histopathological score in DSS-induced murine colitis.

Group	*n*	Weight difference (g)	Colon length (cm)	Colon score
Control	10	1.52 ± 0.68	9.85 ± 1.24	0.18 ± 0.08
DSS	15	−2.36 ± 0.85	6.58 ± 0.99	2.24 ± 0.35

## Data Availability

The datasets used and analyzed during the current study are available from the corresponding author upon reasonable request.
